# ΔNp63 in squamous cell carcinoma: defining the oncogenic routes affecting epigenetic landscape and tumour microenvironment

**DOI:** 10.1002/1878-0261.12473

**Published:** 2019-03-22

**Authors:** Veronica Gatti, Claudia Fierro, Margherita Annicchiarico‐Petruzzelli, Gerry Melino, Angelo Peschiaroli

**Affiliations:** ^1^ Department of Experimental Medicine TOR University of Rome, Tor Vergata Italy; ^2^ Istituto Dermopatico dell'Immacolata IDI‐IRCCS Rome Italy; ^3^ Medical Research Council, Toxicology Unit University of Cambridge UK; ^4^ National Research Council of Italy Institute of Translational Pharmacology Rome Italy

**Keywords:** p63, squamous cell carcinoma, transcription factor, tumour microenvironment

## Abstract

Squamous cell carcinoma (SCC) is a treatment‐refractory tumour which arises from the epithelium of diverse anatomical sites such as oesophagus, head and neck, lung and skin. Accumulating evidence has revealed a number of genomic, clinical and molecular features commonly observed in SCC of distinct origins. Some of these genetic events culminate in fostering the activity of ΔNp63, a potent oncogene which exerts its pro‐tumourigenic effects by regulating specific transcriptional programmes to sustain malignant cell proliferation and survival. In this review, we will describe the genetic and epigenetic determinants underlying ΔNp63 oncogenic activities in SCC, and discuss some relevant transcriptional effectors of ΔNp63, emphasizing their impact in modulating the crosstalk between tumour cells and tumour microenvironment (TME).

**Abbreviations**
APC/C: anaphase‐promoting complex/cyclosome
CSF2: colony stimulating factor 2
DUSP6: dual specificity phosphatase 6
DUSP7: dual specificity phosphatase 7
ECM: extracellular matrix
EGF‐R: epidermal growth factor receptor
EMT: epithelial‐mesenchymal transition
FGF7: fibroblast growth factor 7
FGFR2: fibroblast growth factor receptor 2
HA: hyaluronic acid
HDAC1: histone deacetylases 1
HDAC2: histone deacetylases 2
HNSCC: squamous cell carcinoma of head and neck
HPV: human papilloma viruses
HβD: human beta defensins
IGF‐1: insulin‐like growth factor 1
IGFBP3: IGF binding protein 3
IL: interleukin
IRF6: interferon regulatory factor 6
IRS1: Insulin Receptor Substrate 1
KLF4: transcription factor Krüppel‐like factor 4
MDSCs: myeloid‐derived immunosuppressor cells
MMP9: matrix metalloproteinase 9
NF‐κB: nuclear factor kappa‐light‐chain‐enhancer of activated B cells
NUP62: nucleoporin 62
SCC: squamous cell carcinoma
SRCAP: Snf2‐related CREBBP activator protein
TGFβ2: transforming growth factor‐beta 2
TGFβR2: transforming growth factor beta receptor 2
TGFβ: transforming growth factor beta
TME: tumour microenvironment
VEGF: vascular endothelial growth factor

## 1 Introduction

Squamous cell carcinoma (SCC) is a highly malignant cancer which arises from the squamous epithelium of oesophagus, head and neck, lung and skin. The incidence of SCC varies between different types ranging from 600 000 cases per year for head and neck SCC (HNSCC) to 450 000 cases for lung SCC (Ferlay *et al*., 2015). Although derived from distinct anatomical sites, SCC share a number of unified genomic, clinical and molecular features. The aetiology of SCC is strictly associated with the exposure to several environmental agents (Rothenberg and Ellisen, 2012). The most important risk factors are tobacco use, alcohol consumption and sun exposure. Infection with high‐risk types of human papilloma virus (HPV) has also been associated to the pathogenesis of a subset of HNSCC (Castellsague *et al*., 2016). Intriguingly, HPV‐positive oropharyngeal cancers are associated with a favourable prognosis, likely reflecting the low mutational rate of HPV‐positive tumours (Ang *et al*., 2010).

At clinical level, there is no effective therapy for HNSCC; the therapeutic options include surgery in combination with radiotherapy, chemotherapy or targeted approaches such as epidermal growth factor receptor (EGF‐R) inhibitor (Cetuximab). However, these strategies have not led to a significant increase in the overall 5‐year survival rate, which is approximately 50% for HNSCC patients and 18% for lung SCC (Gillison *et al*., 2015; Sacco and Cohen, 2015). Treatment failure, locoregional recurrence and comorbidities (especially for lung SCC) account for the majority of deaths (Langer *et al*., 2016; Leemans *et al*., 1994; Marur and Forastiere, 2016). In recent years, immune checkpoint inhibitors have been characterized as promising anti‐neoplastic agents in advanced HNSCC, although resistance to the immunotherapy has been observed in most patients *ab initio* (Mehra *et al*., 2018).

At molecular and genetic level, systematic sequencing studies have indicated that frequent genetic and molecular hits dysregulating the activity of two members of the p53 family, p53 itself and p63, are commonly observed in diverse SCC (Agrawal *et al*., 2011, 2012; Cancer Genome Atlas Research Network, 2012; Leemans *et al*., 2018; Pickering *et al*., 2013; Stransky *et al*., 2011). *TP53* gene encodes a transcription factor able to prevent mutations in the genome by promoting cell cycle arrest, DNA repair, metabolic adaptation or apoptosis in response to different stresses (Aubrey *et al*., 2018; Charni *et al*., 2017; Kaiser and Attardi, 2018; Mello and Attardi, 2018; Sullivan *et al*., 2018). For these reasons, p53 is considered the guardian of the genome and its inactivation occurs in the majority of human cancers (Baugh *et al*., 2018; Muller and Vousden, 2013). In SCC, p53 mutation emerges as a dominant early genetic event with a mutational rate of 60–80% of cases and is associated with a more aggressive phenotype (Cancer Genome Atlas, 2015; Poeta *et al*., 2007). Several tumour‐derived p53 mutations are gain‐of‐function mutations and act as driver oncogenes promoting metastatic dissemination and drug resistance (Alexandrova *et al*., 2017; Amelio *et al*., 2018; Kim and Lozano, 2018; Morrison *et al*., 2017; Muller and Vousden, 2014; Parrales *et al*., 2018; Vaughan *et al*., 2017). In addition to gene mutation, others mechanisms may contribute to restraining p53 oncosuppressor activity in SCC, including overexpression/amplification of MDM2, infection with HPV E6 oncoprotein or transcriptional repression by EGF‐R signalling (Kolev *et al*., 2008; Scheffner *et al*., 1990; Wu and Prives, 2018).

In contrast to the high frequency of *TP53* gene mutation, *TP63* gene is rarely mutated in human cancers; rather it is subjected to different genetic and molecular events that either increase its expression or enhance its transcriptional activity (Stransky *et al*., 2011). The relevance of p63 during SCC initiation and progression is supported by studies performed in mouse models of squamous carcinogenesis. The skin‐specific genetic ablation of *TP63* in a mouse model of chemical‐induced skin carcinogenesis induces a rapid and dramatic tumour regression, demonstrating the exquisite dependence of SCC on high levels of p63 (Ramsey *et al*., 2013). In the next paragraphs, we will try to provide a global picture of the oncogenic routes orchestrated by p63, emphasizing the molecular and genetic determinants enhancing its activity in various SCC.

## 2 p63 is a master regulator of epithelial development and homeostasis

p63 is a transcription factor belonging to the p53 family, which includes p53 itself, p63 and p73 (Candi *et al*., 2014; Nemajerova *et al*., 2018). *TP63* gene is expressed as multiple isoforms arising by both alternative promoter usage and differential splicing events at the 3′ end of its RNA. The two main isoforms contain (TAp63) or lack (ΔNp63), the N‐terminal p53‐homologous transactivation domain (Dotsch *et al*., 2010; Yang *et al*., 1998). The ΔNp63α is the most abundant isoform expressed in the basal layer of stratified epithelia, where it maintains the proliferative potential and lineage specification of epithelial structures such as epidermis, lung, thymus and mammary gland (Candi *et al*., 2008; Mills *et al*., 1999; Shalom‐Feuerstein *et al*., 2011; Soares and Zhou, 2018). The critical importance of p63 during epithelial morphogenesis has been demonstrated in diverse animal models and by the functional association of *TP63* mutations with human diseases. Genetic deletion of all p63 isoforms dramatically impairs the development of several epithelial tissues, such as thymus, breast and skin, resulting in premature death because of severe dehydration of the newborns (Mills *et al*., 1999; Yang *et al*., 1999). Notably, the selective genetic deletion of the ΔNp63 isoforms recapitulates the phenotype observed in the p63 global knock‐out mice, strongly indicating that ΔNp63 is the major p63 isoform governing epithelial morphogenesis (Romano *et al*., 2012). In humans, heterozygous mutations in *TP63* cause several developmental disorders, which partially resemble the developmental defects observed in p63 null mice (Celli *et al*., 1999; Rinne *et al*., 2007).

Genome‐wide approaches convincingly established the critical role of p63 in regulating keratinocytes proliferation and differentiation (Kouwenhoven *et al*., 2010, 2015; Rivetti di Val Cervo *et al*., 2012; Truong *et al*., 2006). Recent reports unveiled the key role of ΔNp63 in controlling the epigenetic landscape of epithelial cells, as ΔNp63 recruits epigenetic modulators and chromatin remodelling factors in order to directly regulate numerous target genes involved in cell proliferation, differentiation and adhesion (Fessing *et al*., 2011; Mardaryev *et al*., 2014, 2016).

Based on its critical role in epithelial morphogenesis, it is not surprising that diverse transcriptional and post‐transcriptional mechanisms finely control ΔNp63 expression and activity during squamous differentiation (Lena *et al*., 2008; Rossi *et al*., 2006). Among them, Notch/ΔNp63 cross‐talk is particularly noteworthy, as it regulates the interplay between terminal differentiation and proliferation in squamous epithelia, as well being subjected to distinct oncogenic hits, as we will discuss later (Dotto, 2009; Nguyen *et al*., 2006). In mammals, four NOTCH receptors (NOTCH 1–4) are expressed and synthesized as precursors that undergo specific cleavages in response to ligand interaction. These cleavages release the NOTCH receptor intracellular domain, which translocates to the nucleus and modulates the expression of specific target genes involved in cell fate decisions (Bray, 2006). In the skin, Notch signalling and ΔNp63 activity are functionally interconnected in a finely regulated cross‐talk, which ensures activation of mitogenic and pro‐differentiative signals in distinct epithelial compartments (see Fig. 1, left panel) (Nguyen *et al*., 2006). In the basal layer of epidermis, ΔNp63 inhibits the expression of p21WAF1/Cip1 and HES1, a NOTCH1 target gene, thus sustaining cell cycle progression and repressing late differentiation stages (Nguyen *et al*., 2006; Westfall *et al*., 2003). ΔNp63 is also able directly to induce the expression of the Notch ligand JAG2, likely favouring the initial step of skin differentiation (Candi *et al*., 2007). In the suprabasal layer, NOTCH1 counteracts ΔNp63 activity in a negative feedback loop, directly or through the induction of the interferon regulatory factor 6 (IRF6), which may promote the proteasome‐dependent degradation of ΔNp63 (Moretti *et al*., 2010; Nguyen *et al*., 2006; Thomason *et al*., 2010). Interestingly, in human keratinocytes NOTCH1 expression might also be positively regulated by p53 (Kolev *et al*., 2008; Lefort *et al*., 2007).

**Figure 1:** Schematic diagram of the molecular circuitry connecting squamous differentiation‐related genes in SCC. The genetic alterations of these genes are also reported.

## 3 Genetic determinants of ΔNp63 oncogenic activity in SCC

Over the past years, whole‐exome sequencing has allowed the identification of distinct genetic alterations associated with SCC development. Remarkably, a subset of functionally related genes (*TP63, NOTCH, IRF6*) controlling the squamous differentiation programme is dysregulated in 30–40% of SCC patients. In HNSCC and lung SCC, genomic amplification of the *TP63* locus has been reported in up to 10% and 16% of the cases, respectively (Cancer Genome Atlas Network 2015; Cancer Genome Atlas Research Network, 2012; Pickering *et al*., 2013). In addition, overexpression of ΔNp63 itself is observed in the majority of invasive HNSCC as well as in lung, skin and oesophageal SCC (Agrawal *et al*., 2012; Reis‐Filho *et al*., 2003; Tonon *et al*., 2005). RNA sequencing data indicated that the ΔNp63 isoforms, mainly the α isoform, account for the high expression levels of p63. Indeed, ΔNp63 expression exceeds that of TAp63 more than 200‐fold in lung SCC. These data have been also confirmed in HNSCC cell lines, which express almost exclusively the ΔNp63α isoform (Compagnone *et al*., 2017; Rocco *et al*., 2006). Furthermore, some rare *TP63* mutations reported in HNSCC samples are located in the TA domain, suggesting that ΔNp63 isoform expression is positively selected during tumour evolution (Stransky *et al*., 2011). Collectively, these data indicate that the major p63 isoform driving SCC tumourigenesis is ΔNp63, likely the ΔNp63α isoform (hereinafter referred as ΔNp63).

The relevance of ΔNp63 during SCC initiation and progression is also supported by studies performed in mouse models. The induction of moderate expression of ΔNp63 in the basal layer of stratified epithelia indeed causes the development of spontaneous epidermal cysts that resemble cutaneous premalignant lesions (Devos *et al*., 2017). Furthermore, in a model of chemical‐induced skin carcinogenesis, ΔNp63 expression accelerates the onset of papilloma occurrence, suggesting that ΔNp63 favours the early steps of SCC development (Devos *et al*., 2017).

In addition to gene amplification and/or overexpression, other genetic alterations foster ΔNp63 oncogenic activity in SCC. As stated before, Notch signalling is fundamental for the proper squamous epithelia homeostasis. In SCC, diverse genetic events dysregulate the Notch/ΔNp63 crosstalk. *NOTCH1* point mutations occur in 11–15% of HNSCC, in 8% of lung SCC and in more than 40% of cutaneous SCC (Agrawal *et al*., 2011, 2012; Pickering *et al*., 2013). Point mutations in the *NOTCH2* gene have been also reported in 11% of HNSCC samples; these mutations are mutually exclusive and exhibit minimal overlap with amplification of the *TP63* gene (Stransky *et al*., 2011). These observations suggest that aberrations in squamous differentiation modulators, which act in the same functional axis, have overlapping functional consequences. Importantly, *NOTCH* mutations are loss‐of‐function, missense or nonsense mutations, a strong indication of a tumour‐suppressive function of Notch signalling in SCC. This conclusion is also supported by *in vivo* evidence showing that *Notch1* inactivation in the mouse epidermis promotes skin tumourigenesis (Nicolas *et al*., 2003; Proweller *et al*., 2006). In addition to gene mutation, NOTCH activity is also restrained by the inhibitory action of ΔNp63 itself (see section ‘Genetic determinants of ΔNp63 oncogenic activity in SCC’). Furthermore, the high rate of *TP53* mutation and the frequent amplification of *EGF‐R* locus in SCC may cooperate to maintain the low expression of NOTCH1, thus favouring tumour proliferation (Kolev *et al*., 2008).

As anticipated, another squamous differentiation‐related gene functionally connected with the Notch signalling and ΔNp63 is *IRF6*. *IRF6* encodes for a transcription factor, acting as an important mediator of the Notch pro‐differentiation function. The Notch signalling sustains the expression of IRF6, which contributes to the activation of growth/differentiation‐related genes (Nguyen *et al*., 2006). At the same time IRF6 is able to restrain ΔNp63 protein levels by enhancing its protein degradation (Moretti *et al*., 2010). Diverse genetic events such as promoter methylation and gene mutation impair IRF6 activity in SCC (Rotondo *et al*., 2016). Mutations of the *IRF6* gene have been reported in 7% of HNSCC patients and down‐regulation of IRF6 has been correlated with tumour invasive and differentiation status of SCC (Stransky *et al*., 2011).

Genomic amplification or overexpression of another squamous differentiation‐related gene, *SOX2*, also contribute to enhance and activate ΔNp63 oncogenic activity. The *SOX2* gene lies approximately 10 Mb from *TP63,* and it is frequently amplified in lung, oesophageal and oral SCC (Ferone *et al*., 2016; Zhou *et al*., 2017). SOX2 and ΔNp63 proteins physically interact and exhibit overlapping genomic occupancy at a large number of loci in SCC, enhancing the expression of pro‐survival factors (Jiang *et al*., 2018; Watanabe *et al*., 2014).

Collectively, these data suggest that distinct genetic events, such as *NOTCH* mutations, *TP63* genomic amplification/overexpression, *TP53* mutation, IRF6 down‐modulation and SOX2 amplification (see Fig. 1, right panel), may promote an immature and more proliferative basal‐like phenotype by, at least in part, fostering ΔNp63 oncogenic activity.

## 4 Deregulation of factors controlling ΔNp63 levels and activity in SCC

In addition to these genetic lesions, SCC exhibits transcriptional alterations of factors involved in controlling ΔNp63 expression at both mRNA and protein level. One well‐established example is represented by ASPP2, a member of the ASPP family of proteins, which is able to repress ΔNp63 expression through a nuclear factor kappa‐light‐chain‐enhancer of activated B cells (NF‐κB)‐dependent mechanism (Tordella *et al*., 2013). Down‐regulation of ASPP2 is frequently observed in human HNSCC and is associated with increased p63 expression. Notably, *Tp63* is required for the development of spontaneous SCC observed in ASPP2^−/+^ BALB/c heterozygous mice, implicating p63 as a critical mediator of ASPP2 tumour‐suppressive function in SCC (Tordella *et al*., 2013).

ΔNp63 levels can be also modulated by post‐transcriptional mechanisms, mainly by ubiquitin‐mediated proteolysis. Several E3 ubiquitin ligases targeting ΔNp63 have been identified so far, e.g. RACK1, NEDD4, ITCH, FBW7 and WWP1, each of them likely contributing to modulate ΔNp63 protein levels in tumours (Bakkers *et al*., 2005; Fomenkov *et al*., 2004; Galli *et al*., 2010; Li *et al*., 2008; Malatesta *et al*., 2013; Peschiaroli *et al*., 2010; Rossi *et al*., 2006). For instance, *FBW7* is a tumour‐suppressor gene frequently mutated in a variety of solid tumours, including SCC of different origins (Xiao *et al*., 2018). Recently, Prives’s group has identified the anaphase‐promoting complex/cyclosome (APC/C) as a novel E3 ligase triggering ΔNp63 degradation in mitosis and during terminal differentiation (Rokudai *et al*., 2018). Although further studies are necessary to provide formal proof of the involvement of this degradative pathway in SCC development, some observations favour this conclusion. In detail, a ΔNp63 mutant refractory to APC/C activity increases keratinocyte proliferation, inhibits differentiation and has oncogenic activity in xenograft tumour transplantation assays. More importantly, high levels of STXBP4, a factor counteracting APC/C‐mediated ubiquitination of ΔNp63, significantly correlate with the accumulation of ΔNp63 in skin and lung SCC (Rokudai *et al*., 2018). However, this correlation might also result from the inhibitory effect exerted by STXBP4 on diverse ΔNp63 targeting E3 ligases, such as ITCH and RACK1 (Li *et al*., 2009).

Another recent report unveils a novel mechanism which can contribute to sustain ΔNp63‐mediated transcriptional activity in SCC. Hazawa *et al*. reported that nucleoporin 62 (NUP62) promotes ΔNp63 nuclear localization in SCC. NUP62 is highly expressed in stratified squamous epithelia and its abundance is further increased in SCC, thus maintaining elevated nuclear ΔNp63 levels (Hazawa *et al*., 2018).

In conclusion, these data clearly indicate that distinct genetic and molecular events foster ΔNp63 activity in SCC, strengthening the concept that ΔNp63 oncogenic activity is of critical importance for SCC initiation and progression.

## 5 Transcriptional effectors of ΔNp63 oncogenic function in SCC

Initially, it was hypothesized that the oncogenic role of ΔNp63 in SCC mainly relies on its ability to act as a dominant‐negative factor to p53/p73 proteins and repress their ability to activate the expression of target genes involved in apoptosis or cell cycle (DeYoung *et al*., 2006; Rocco *et al*., 2006; Westfall *et al*., 2003; Yang *et al*., 1998). In HNSCC cells, it has been showed that ΔNp63 is able to interact with p73, restraining the transcriptional activation of the pro‐apoptotic gene *PUMA*. Accordingly, down‐modulation of p63 relieves p73 and induces cell death, a phenomenon reversed by the overexpression of BCL‐2, an important anti‐apoptotic protein (Adams and Cory, 2018; Kale *et al*., 2018; Strasser and Vaux, 2018). Although this mechanism may be relevant for the pro‐survival effect exerted by ΔNp63, other observations suggested alternative molecular mechanisms by which ΔNp63 exerts its oncogenic function in SCC. First, ΔNp63 protein is able to transactivate specific target genes due to the presence of two transactivation domains, one located between the oligomerization domain and the SAM domain, and another at the first 26 amino acids (Dohn *et al*., 2001; Ghioni *et al*., 2002; Helton *et al*., 2006; Lena *et al*., 2015). Secondly, in lung SCC and HNSCC, ΔNp63 acts as a potent transcriptional repressor and diverse epigenetic factors have been implicated in ΔNp63‐mediated transcriptional repression. Thirdly, most SCC exhibits both overexpression of ΔNp63 and inactivating mutations in *TP53*, suggesting the existence of p53‐independent oncogenic functions of ΔNp63 (Neilsen *et al*., 2011; Nekulova *et al*., 2011). Last but not least, in p53 wild‐type lung SCC cells, depletion of p53 or p73 does not rescue the proliferation arrest caused by ΔNp63 knockdown (Gallant‐Behm *et al*., 2012). Collectively, these observations clearly indicate that the activation or repression of diverse transcriptional target genes is a critical oncogenic outcome of ΔNp63 activity in SCC, even though some transcriptional independent mechanisms have been described (Patturajan *et al*., 2002). Below, we will describe the transcriptional effectors of ΔNp63 oncogenic activity, emphasizing their role in controlling tumour proliferation, survival and dissemination.

### 5.1 ΔNp63‐repressed genes in SCC

The genesis and homeostasis of stratified epithelia, such as the epidermis, require the coordinated regulation of proliferation, adhesion, migration and differentiation. During the initiation and progression of SCC the fine balance between these processes is altered. Generally, SCC cells exhibit increased proliferative capabilities at the expense of a diminished ability to undergo the terminal differentiation programme. Probably one of the most important ΔNp63‐repressed genes involved in controlling the proliferation‐differentiation crosstalk is *NOTCH1*.

As we described before, ΔNp63 is able to inhibit Notch signalling mainly by transcriptional repression of the *HES1* gene, a downstream target of NOTCH1. In addition to this indirect mechanism, a direct transcriptional effect of ΔNp63 on *NOTCH1* gene expression has been also observed (Yugawa *et al*., 2010). In diverse normal and SCC cells, ΔNp63 may directly repress the transcription of *NOTCH1* gene through a p53‐responsive element. Interestingly, the ability of ΔNp63 to affect NOTCH1 expression negatively has also been observed in the epidermis of ΔNp63 knock‐out mouse embryos (Romano *et al*., 2012), suggesting that the ΔNp63/NOTCH1 pathway might be indicative of a regenerative state of tumour cells. The ΔNp63‐mediated repression of NOTCH1 has two major consequences: it inhibits the NOTCH1‐mediated activation of terminal differentiation programme and sustains cell proliferation by suppressing the expression of the cyclin‐dependent kinase (CDK) inhibitor p21WAF1/Cip1. ΔNp63 may also repress p21WAF1/Cip1 expression directly (Westfall *et al*., 2003) or through an NF‐κB‐dependent mechanism (Nguyen *et al*., 2006) .

Another ΔNp63‐repressed gene involved in finely regulating the proliferation/differentiation crosstalk is the transcription factor Krüppel‐like factor 4 (KLF4). KLF4 is a key driver of squamous differentiation and is highly expressed in differentiating both oesophageal epithelial cells and keratinocytes, which, in cooperation with ZNF750, drives the commitment to terminal differentiation (Boxer *et al*., 2014; Sen *et al*., 2012). ΔNp63 is able directly to repress KLF4 transcription and enhance ZNF750 expression to activate an early step of squamous differentiation (Cordani *et al*., 2011; Sen *et al*., 2012). However, ZNF750 can also induce KLF4 expression (Sen *et al*., 2012), suggesting a complex interplay between ΔNp63 and effectors of early and terminal differentiation. Although it is not clear whether KLF4 and ZNF750 represent critical effectors of ΔNp63 oncogenic activity in SCC, several observations suggest their tumour‐suppressive function. Genetic ablation of *KLF4* in the oesophagus results in delayed differentiation and development of precancerous squamous cell dysplasia (Tetreault *et al*., 2010). KLF4 is downregulated in human oesophageal squamous cell carcinoma (Luo *et al*., 2004; Wang *et al*., 2002) and *KLF4* loss also promotes skin carcinogenesis in mice (Li *et al*., 2012). Down‐modulation of ZNF750 activity by gene mutation, deletion or under‐expression has been observed in human SCC, and low ZNF750 expression is associated with poor survival (Hazawa *et al*., 2017; Zhang *et al*., 2018). These data indicate that the ΔNp63/KLF4/ZNF750 axis might be important in the prevention of terminal differentiation and promotion of SCC tumourigenesis.

More recently, Ellisen's group has identified another ΔNp63 oncogenic pathway, which fine‐tunes the proliferation/differentiation crosstalk in SCC (Saladi *et al*., 2017). By comparing ChIP‐seq and RNA‐seq data in normal versus HNSCC cells, these authors have identified a tumour‐specific transcriptional profile directly regulated by ΔNp63. Notably, the expression of the majority of direct ΔNp63 target genes is upregulated in response to ΔNp63 silencing, indicating the dominant function of ΔNp63 as transcriptional repressor in SCC. *WWC1* (*KIBRA*) is one of the top genes repressed by ΔNp63 in HNSCC. WWC1 encodes a cytosolic phosphoprotein that acts as a potent regulator of the Hippo pathway by favouring YAP cytoplasmic retention (Furth and Aylon, 2017; Yu *et al*., 2010; Zhao *et al*., 2007). By repressing the transcription of WWC1, ΔNp63 favours YAP nuclear activity, thereby promoting proliferation and inhibiting differentiation. As we will discuss later, HNSCC frequently displays amplification of ACTL6a, an epigenetic factor necessary for the ΔNp63‐mediated repression of WWC1.

The critical relevance of the ΔNp63‐mediated transcriptional repression in SCC evolution has also been highlighted by the identification of diverse ΔNp63‐negative target genes acting as key players of cell proliferation control in lung SCC. IGF binding protein 3, IGFBP3, is noteworthy, as its transcriptional control has been previously linked to the activity of p53 family members. The p53 activation is able to enhance the secretion of an active form of IGFBP3 which is capable of inhibiting mitogenic signalling by the insulin‐like growth factor IGF‐1 (Buckbinder *et al*., 1995). However, the p53‐dependent transactivation of IGFBP3 appears to be cell type‐specific, as in the H226 cell line, p53 activation does not lead to IGFBP3 induction (Gallant‐Behm *et al*., 2012). Conversely, in several SCC cells, IGFBP3 expression is under the negative control of ΔNp63, through an H2A.Z‐mediated transcriptional repression (Barbieri *et al*., 2005; Gallant‐Behm *et al*., 2012). Furthermore, diverse data have indicated that ΔNp63‐dependent regulation of IGFBP3 might be important for SCC progression. ΔNp63 and IGFBP‐3 expression are inversely correlated in human SCC samples and decreased IGFBP3 expression is correlated with unfavourable prognosis in human cancers (Barbieri *et al*., 2005; Chang *et al*., 2002; Katsaros *et al*., 2001), implying a potential relevance of IGFBP3 suppression in SCC development.

More recently, Espinosa's group has exploited a genome‐wide CRISPR‐Cas9 screen to identify the pathway required for the ΔNp63‐driven proliferation in lung SCC (Abraham *et al*., 2018). Upon ΔNp63 silencing, lung SCC cells undergo a block of proliferation which is dependent on the activation of the transforming growth factor beta (TGFβ) signalling. At molecular level, ΔNp63 directly represses the transcription of TGFB2 and TGFBR2, thus restraining the activation of the TGFβ signalling. Interestingly, the cell cycle arrest mediated by ΔNp63 silencing is also dependent on the expression of RHOA, a small GTPase activated by TGFβ signalling and commonly down‐regulated in lung SCC specimens. Although these data unveil a novel ΔNp63 oncogenic pathway controlling lung SCC proliferation, they do not address its effect in p53 mutated background. This is quite important, as the majority of SCC harbour mutations in the *TP53* locus and TGFβ signalling can exert tumour‐prone or tumour‐suppressive effects depending on cell context as well as on the p53 status (Ikushima and Miyazono, 2010; Karlsson *et al*., 2017). Interestingly, the dependence on RHOA to sustain cell cycle arrest upon ΔNp63 depletion has not been observed in the immortalized keratinocyte cell line HaCaT, which harbours mutation of *TP53* gene (Abraham *et al*., 2018). Furthermore, in HNSCC cells, ΔNp63 can enhance the pro‐tumourigenic function of TGFβ by repressing the expression of two microRNA (miRNA), miR‐527 and miR‐665, which target Smad4 and TGFβR2, respectively (Rodriguez Calleja *et al*., 2016). Therefore, the effect of ΔNp63 on TGFβ signalling might be cell context‐dependent and/or influenced by extrinsic factors, as we will discuss later.

In addition to miR‐527 and miR‐665, ΔNp63 can activate or repress the expression of diverse miRNA involved in a variety of tumour‐related processes (Lin *et al*., 2015; Ory *et al*., 2011; Ratovitski, 2013). However, the involvement of the ΔNp63‐miRNA pathway in SCC pathogenesis is not well characterized and our knowledge of its actions as critical effectors of ΔNp63 oncogenic activity is quite limited.

### 5.2 Epigenetic determinants of ΔNp63‐mediated transcriptional repression in SCC

In the past years, diverse molecular mechanisms underlying ΔNp63‐mediated transcriptional repression have been elucidated (see Fig. 2). The general picture is that ΔNp63 binds to and employs as co‐repressor several chromatin remodelling factors. In HNSCC, ΔNp63 can form a complex with the histone deacetylases HDAC1 and HDAC2 (Ramsey *et al*., 2011). HDACs mediate transcriptional regulation by increasing histone‐DNA affinity, thus promoting the formation of a chromatin‐condensed structure that prevents transcription factor binding (Li and Seto, 2016; Paluvai *et al*., 2018). ΔNp63 exploits this mechanism mainly for repressing pro‐apoptotic genes such as *PUMA*, then favouring cell survival. This anti‐apoptotic pathway can be disrupted by chemotherapeutic agents such as cisplatinum, which displace the HDAC/ΔNp63 complex from the *PUMA* promoter, thus favouring its expression and triggering, as a consequence, apoptosis. This pro‐survival mechanism may inhibit the treatment of p63 overexpressing cells with the HDAC inhibitors trichostatin A (TSA) and Vorinostat. Remarkably, HNSCC cell lines show a direct correlation between ΔNp63 protein levels and TSA sensitivity (Ramsey *et al*., 2011), and increased expression of HDAC is frequently observed in SCC where it predicts poor patient prognosis (Chang *et al*., 2009; Theocharis *et al*., 2011). This evidence supports the rationale of several ongoing clinical trials, which are coupling HDAC inhibitors with conventional chemotherapy for SCC treatment (Caponigro *et al*., 2016; Teknos *et al*., 2018).

**Figure 2:** Model of the epigenetic mechanisms exploited by ΔNp63 to repress transcription in various SCC. (A) In HNSCC cells, ΔNp63 may recruit the histone deacetylates HDAC1 and HDAC2 to chromatin, preventing transcription factor binding to the promoters of pro‐apoptotic genes, such as *PUMA*. (B) In lung SCC cells, ΔNp63 is able to repress the transcription of anti‐proliferative genes by promoting H2A.Z incorporation. (C) In HNSCC cells, ΔNp63 interacts with the SWI/SNF subunit ACTL6A, inducing the repression of anti‐proliferative genes.

It is worth noting that the molecular mechanisms exploited by ΔNp63 to repress its target genes might be dependent on cell context (Gallant‐Behm *et al*., 2012). Indeed, in H226 cells, ΔNp63 represses the expression of its targets independently from HDAC action. In this lung SCC cell line, ΔNp63 takes part in a large chromatin remodelling protein complex called SRCAP that is able to exchange histone H2A with the histone variant H2A.Z and may act as a transcriptional repressor when arranged near the transcription start sites (Marques *et al*., 2010). H2A.Z deposition is involved in the repression of several ΔNp63 target genes such as *ZHX2*,* NTN4*,* SAMD9L* and *IGFBP3*, each of them likely contributing to the ΔNp63‐mediated control of cell proliferation (Gallant‐Behm *et al*., 2012).

More recently, the SWI/SNF complex has been involved in ΔNp63‐mediated transcriptional repression in HNSCC (Saladi *et al*., 2017). SWI/SNF is a multisubunit chromatin remodelling complex that catalyses nucleosome sliding or ejection, modulating DNA accessibility to the transcription machinery (Patel and Vanharanta, 2016; Wilson and Roberts, 2011). In HNSCC, ΔNp63 interacts with the SWI/SNF subunit ACTL6A, inducing the repression of WCC1 transcription, as we have described before. In contrast to what is observed in normal stratified epithelium, *ACTL6A* is frequently overexpressed in HNSCC and about 20% of HNSCC shows genomic co‐amplification of *ACTL6A* and *TP63* loci (Saladi *et al*., 2017). Furthermore, elevated levels of ACTL6A expression are a negative prognostic factor of HNSCC patient survival, suggesting that ACTL6A has an oncogenic function in HNSCC (Saladi *et al*., 2017). Conversely, in different types of cancer, genomic analysis identified several loss‐of‐function mutations in various SWI/SNF subunits, suggesting a tumour‐suppressor role for this complex (Kadoch *et al*., 2013). This apparent contradiction can be mechanistically explained, taking into account that in epidermal progenitor cells, ACTL6A contributes to maintain the undifferentiated state preventing SWI/SNF complex, by binding and transactivating differentiation genes (Bao *et al*., 2013).

These molecular data together with the key importance of ΔNp63‐repressed pathways in mediating the mitogenic action of ΔNp63 in SCC clearly indicate that ΔNp63‐mediated transcriptional repression is a crucial oncogenic outcome of ΔNp63 in SCC as well as in other epithelial cancers (Regina *et al*., 2016a,2016b). On the other hand, as described in the next paragraph, ΔNp63 also exerts its oncogenic activity by enhancing the transcription of several pro‐tumourigenic factors, and epigenetic modifications are likely to be involved in this oncogenic function. Accordingly, a high mutation rate of the methyltransferase KMTD2, an ΔNp63 interacting epigenetic factor involved in the transcriptional activation of epithelial target genes, has been observed in SCC (Lin‐Shiao *et al*., 2018). Deciphering the global epigenetic landscape regulated by ΔNp63 and its involvement in SCC tumourigenesis needs to be fully explored and represents an important direction for future studies.

### 5.3 Oncogenic routes activated by ΔNp63 in SCC

Besides acting as a transcriptional repressor, ΔNp63 enhances the transcription of diverse pro‐tumourigenic genes playing a critical role in SCC tumourigenesis. Remarkably, a significant group of ΔNp63‐positive target genes codifies for proteins related to extracellular matrix (ECM) or involved in the growth factor‐mediated signalling (see Fig. 3). In the following sections, we will describe some of these ΔNp63‐activated genes, emphasizing their role in modulating the crosstalk of tumour cells, ECM and tumour microenvironment (TME).

**Figure 3:** Schematic model of the ΔNp63 oncogenic routes in SCC. The green and red arrows indicate the pathways under positive and negative regulation by ΔNp63, respectively. See text for details.

#### 5.3.1 ECM‐mediated signalling

The initial observations that ΔNp63 might actively participate in modulating the composition of ECM and activate ECM‐mediated signalling were reported in non‐transformed cells. In normal mammary epithelial cells, silencing of p63 induces cell detachment and anoikis, and the concomitant modulation of the expression of several adhesion molecules and ECM receptors. ΔNp63 enhances the expression of integrin receptors (e.g. ITGB1, ITGB4, ITGA6, ITGA3), ECM components such as laminin and collagen (e.g LAMC2 and COL17A1) and adhesion molecules (e.g. PERP and ZNF185) (Carroll *et al*., 2006; Ihrie *et al*., 2005; Kurata *et al*., 2004; Smirnov *et al*., 2019).

Although a formal demonstration that these ECM‐related factors are required for ΔNp63 oncogenic function in SCC is missing, several data indicate that they may significantly participate in SCC development. Tumour regression upon *TP63* excision is associated with decrease of expression of ECM‐related proteins, such as collagen COL6A2 and COL17A1, LAMB3 and ITGB4 (Ramsey *et al*., 2013). In line with this evidence, the integrin‐mediated adhesion and signalling is one of the tumour‐specific programmes regulated by ΔNp63 in HNSCC cell lines (Saladi *et al*., 2017). Furthermore, increased suprabasilar expression of α6β4‐integrin occurs in more than 70% of HNSCC with higher invasive‐metastatic potential (Van Waes *et al*., 1995). Together with the pro‐tumourigenic pathway exerted by ITGB4/EGF‐R signalling crosstalk (Carroll *et al*., 2006), these data suggest that ECM‐mediated signalling might be functionally important during SCC development.

In agreement with this, our group has recently unveiled a novel ΔNp63‐dependent transcriptional oncogenic programme aimed at sustaining the synthesis of one important component of the ECM, hyaluronic acid (HA) (Compagnone *et al*., 2017). In human tumours, HA is pivotal for diverse tumour‐related processes, including cell migration, angiogenesis and metastasis (Chanmee *et al*., 2016; Jiang *et al*., 2011; Toole, 2004), and several types of cancers including SCC are characterized by relatively high amounts of tumour cell‐associated HA (Koyama *et al*., 2007, 2008; Kultti *et al*., 2014). We have demonstrated that ∆Np63 is able to drive the expression of the HA synthase gene *HAS3* and the HA receptor CD44, thus favouring the HA/CD44‐mediated oncogenic signaling in HNSCC. In detail, ΔNp63 favours the activation of pro‐mitogenic and pro‐survival signals by EGF‐R in an HA‐dependent manner. Interestingly, EGF‐R expression has been positively correlated with that of HAS3 in human oesophageal SCC tumours (Twarock *et al*., 2011) and activation of EGF‐R enhances HAS3 expression in some tumour cells (Bourguignon *et al*., 2007; Chow *et al*., 2010), implying a positive feedback between EGF‐R signalling and ∆Np63‐HAS3 pathway in HNSCC. The functional importance of the ∆Np63‐mediated regulation of HA signalling in human tumours is highlighted by diverse observations. In HNSCC tumours, p63 expression is positively correlated with that of HAS3 and CD44, and the expression of three tumour‐related CD44 variants is associated with HNSCC progression in clinical samples (Maula *et al*., 2003; Misra *et al*., 2011). More importantly, high expression of *TP63/HAS3* axis is a negative prognostic factor of HNSCC patient survival, indicating that the functional link between ΔNp63 and HA/CD44 signalling critically contributes to HNSCC progression and therapeutic response (Compagnone *et al*., 2017). Although these data reveal a novel ∆Np63 oncogenic route in HNSCC, further studies will be necessary to understand whether HA synthesis inhibition could be exploited as a novel therapeutically actionable pathway in HNSCC.

#### 5.3.2 Growth factor‐mediated signalling

In addition to ECM‐related proteins, ∆Np63 controls the expression of ligands, receptors and intracellular mediators of diverse growth factors, thus favouring the activation of pro‐survival and mitogenic signals. One important example of such regulation is related to the activation of EGF‐R signalling. EGF‐R amplification has been observed in many SCC and its expression has been correlated with poor outcome (Chung *et al*., 2006; Ozawa *et al*., 1987; Sigismund *et al*., 2018; Temam *et al*., 2007; Wintergerst *et al*., 2018). The overall survival rate and time of relapse of HNSCC patients overexpressing EGF‐R is significantly shorter than those without EGF‐R overexpression. At the clinical level, anti‐EGFR monoclonal antibody (cetuximab) in combination with radiation or chemotherapy is currently approved as a targeted therapy for the treatment of selected HNSCC patients, even if gain of EGFR has not been clearly demonstrated to be predictive for the outcomes following cetuximab therapy (Bonner *et al*., 2006; De Pauw *et al*., 2018; Licitra *et al*., 2011).

∆Np63 oncogenic activity participates in sustaining EGF‐R‐mediated signalling by activating distinct pathways. In diverse epithelial tumours, ∆Np63 directly activates the transcription of EGF‐R, even though this mechanism seems to be tissue‐specific (Danilov *et al*., 2011). ∆Np63 is also able to induce the transcription of neuregulin (NRG1), a natural ligand of ErbB3 receptor (Forster *et al*., 2014). In HNSCC, full EGF‐R activation is dependent on the ErbB3‐neuregulin axis. (Redlich *et al*., 2018). Compared with other tumours, HNSCC have among the highest levels of NRG1, and tumours recurrence further increases neuregulin‐1 expression after curative treatments with radiation and chemotherapy (Wilson *et al*., 2011). In addition to transcriptional activation of these EGFR‐related factors, ∆Np63 might also sustain EGF‐R signalling by regulating the expression of ECM‐related factors, such as ITGB4, HA and CD44. Collectively, these data indicate that ∆Np63 exploits multiple oncogenic pathways to enhance EGF‐R‐mediated oncogenic signalling.

A recent report connected ∆Np63 transcriptional activity with the activation of another receptor tyrosine kinase, the insulin growth factor receptor 1 (IGFR‐1). In HNSCC cell lines ∆Np63 positively controls the transcription of the adaptor protein Insulin Receptor Substrate 1 (IRS1), an important mediator of the pro‐survival and mitogenic signalling of insulin and IGF‐1 (Frezza *et al*., 2018). The modulation of IRS1 levels by ∆Np63 is interesting in light of the role of ∆Np63 in preventing the expression of IGFBP3, which regulate the bioavailability and half‐life of circulating IGF‐1 (Barbieri *et al*., 2005). By repressing IGFBP3 and concomitantly activating IRS1 expression, ∆Np63 is able to enhance circulating IGF‐1 and increase its intracellular signalling, ultimately fostering the growth and survival of SCC cells. However, further studies are needed to clarify the clinical impact of the ∆Np63/IGF signaling, as contradictory findings on the prognostic impact of IGF signalling have been reported in HNSCC (Dale *et al*., 2015; Lara *et al*., 2011; Luo *et al*., 2014; Sun *et al*., 2011).

The regulation of the expression of FGF‐R2, a member of the fibroblast growth factor (FGF) receptor family, is another example of how ∆Np63 controls growth factor‐mediated signalling. *In vitro* and *in vivo* evidence demonstrated that FGF‐R2 is a relevant ∆Np63 transcriptional target gene exerting a pro‐tumourigenic signalling in SCC (Ramsey *et al*., 2013). Remarkably, activation of FGF‐R2 requires stromal‐dependent secretion of FGF7, the most specific ligand for FGF‐R2 (Wesche *et al*., 2011), resulting in a specific and spatial activation of FGF‐R2 signalling in tumour cells. Besides revealing a novel ∆Np63‐driven oncogenic pathway with a potential therapeutic impact, these data uncovered a functional link between ∆Np63 activity and tumour stroma interaction. In the next section, we will expand this concept by reporting a few examples of the interplay between ∆Np63 transcriptional activity and TME in SCC.

#### 5.3.3 TME‐related signalling

Tumour development likely arises by the co‐evolution of tumour cells and cellular components of the stroma. The close relationship between tumour cells and the stroma is fundamental for adapting and modifying TME to sustain and enhance tumour growth and invasion (Bissell and Radisky, 2001; Junttila and de Sauvage, 2013; Schaaf *et al*., 2018). Stromal components include different types of cells, including cancer‐associated fibroblasts (CAF), endothelial cells and infiltrating immune cells. Tumour stroma interaction likely generates an intricate network of signals that significantly sustains the development of different types of cancer, and SCC is not an exception. HNSCC and other squamous carcinomas are characterized by a tight interaction of malignant cells with a dense fibrous stroma, and high levels of stromal infiltrate are associated with poor prognosis in SCC (Fujii *et al*., 2010; Takahashi *et al*., 2011).

Few data have established a functional link between ∆Np63 oncogenic activity and changes of the TME. By recruiting two NF‐κB family members, cRel and RelA, ∆Np63 co‐regulates a subset of pro‐inflammatory cytokines, such as interleukin (IL)‐1, IL‐6, IL‐8 and colony stimulating factor 2 (CSF2) (Yang *et al*., 2011). These pro‐inflammatory factors are known to attract infiltrating neutrophils and macrophages, and individually are known to promote the aggressive malignant behaviour that leads to poor prognosis of HNSCC (Allen *et al*., 2007; Chen *et al*., 1999). In human HNSCC samples and in ΔNp63 transgenic mice, ΔNp63 levels are correlated with the presence of infiltrating inflammatory cells (Yang *et al*., 2011). Interestingly, increased ΔNp63 expression and inflammatory cell infiltration in oral leukoplakias are associated with worse prognosis and higher rate of cancer progression (Saintigny *et al*., 2009).

By recruiting neutrophils and macrophages, ΔNp63 might also sustain tumour‐associated angiogenesis. In osteosarcoma cells, ectopic expression of ΔNp63 induces VEGF secretion by activating STAT3/HIF‐1α pathway in a cytokine‐dependent manner (Bid *et al*., 2014). Although this pro‐angiogenic pathway has not been formally proved to occur in SCC, another report suggested a link between ΔNp63 and lymphoangiogenesis in SCC. ΔNp63 enhances the transcription of three human beta defensins (HβD1, HβD2 and HβD4), a class of antimicrobial peptides secreted in inflammatory conditions by epithelial cells (Suarez‐Carmona *et al*., 2014). By doing this, ΔNp63 stimulates the migration of lymphatic endothelial cells in a CCR6‐dependent manner, which might explain the increased density of blood and lymphatic vessels observed in high ΔNp63‐expressing SCC.

Recent evidence in other epithelial tumours also confirmed a functional role of ΔNp63 in modelling TME. In triple negative breast cancer (TNBC) cells, ΔNp63 drives the recruitment of myeloid‐derived immunosuppressor cells (MDSCs) by direct activation of the chemokines CXCL2 and CCL22 (Kumar *et al*., 2018). Importantly, MDSCs secrete pro‐metastatic factors, such as MMP9 and chitinase 3‐like 1, which in turn promote TNBC tumour progression and metastasis.

These data indicate that ΔNp63‐activated pathways may modify TME to create a favourable niche for tumour progression. On the other hand, it is reasonable that TME could also influence ΔNp63 oncogenic activity. Although this relationship is far to be fully explored, there are a few indications that TME might be a critical determinant in controlling the biological outcome of ΔNp63 activity. The role of TGFβ in determining the pro‐migratory and pro‐invasive function of ΔNp63 is an example of the critical impact of TME on ΔNp63 oncogenic function. Several reports have ascribed opposite functions to ΔNp63 in controlling tumour dissemination in diverse tumour types, including SCC (Cho *et al*., 2010; Giacobbe *et al*., 2016; Wu *et al*., 2014). Generally, it has been established that the anti‐metastatic action of ΔNp63 in squamous tumours relies on its ability to maintain the epithelial identity and repress mesenchymal traits, thus inhibiting the EMT process. ΔNp63 deregulates the expression of several genes, such as *POSTN*,* CDH2*,* L1CAM* and *WNT5A*, which contributes to the anti‐migratory ability exerted by p63 in SCC (Barbieri *et al*., 2006). Conversely, other data have suggested a pro‐tumourigenic effect of ΔNp63 on tumour dissemination. Exogenous ΔNp63 can enhance the migration rate of oesophageal squamous carcinoma cells (Lee *et al*., 2014) and ΔNp63 is required for HNSCC cancer cell migration as well (Yang *et al*., 2011). Although these conflicting results might be ascribed to different experimental approaches or different cellular models, it is also possible that extrinsic factors could be determinant in regulating the outcome of ΔNp63 on cell migration and invasion. Accordingly, several reports have indicated in the TGFβ pathway a parameter controlling this ΔNp63 oncogenic function. In a TGFβ‐rich environment, osteosarcoma cells display increased motility and metastatic dissemination upon overexpression of ΔNp63 (Rodriguez Calleja *et al*., 2016). In SCC cells, TGFβ signalling activates ΔNp63 transcriptional activity, which in turn induces the transcription of two direct target genes, *DUSP6* and *DUSP7* (Vasilaki *et al*., 2016). Ablation of ΔNp63 or DUSP6/7 perturbs the TGFβ‐induced migration and invasion. Although the proposed molecular mechanism underlying the TGFβ‐dependent activation of ΔNp63 activity has not been fully clarified, these data suggest that TME could critically contribute to determine the oncogenic function of ΔNp63.

Other observations in different epithelial tumours further support this hypothesis. Basal‐like breast cancer cells that express ΔNp63 rely on mammary fibroblasts to initiate ECM reorganization, permiting collective invasion (Dang *et al*., 2011, 2015). Similarly, luminal B type breast cancer cells expressing ΔNp63 are limited to invading regions enriched in collagen I (Cheung *et al*., 2013). These data suggest that changes of TME during tumour evolution might be of extreme importance in the fine regulation of ΔNp63 oncogenic activity.

## 6 Concluding remarks

Squamous cell carcinoma is a highly malignant cancer and the therapeutic options have not led to a significant increase in the overall survival rate. A common feature of SCC of diverse epithelial origins is their dependence on the oncogenic function of the transcription factor ΔNp63. A variety of ΔNp63 transcriptional target genes involved in the regulation of cell adhesion, growth factor signalling, migration and invasion have been identified, and, presumably, each of them contributes to the positive regulation of SCC development. At the molecular level, ΔNp63 exerts its oncogenic function by recruiting distinct epigenetic factors, mainly transcriptional repressor complexes. ΔNp63 acts also as transcriptional activator and it is reasonable that these two opposite functions of ΔNp63 must be finely regulated during SCC initiation and progression. It would be intriguing to assess whether changes of the ΔNp63‐dependent epigenetic landscape are functionally linked to the different stages of SCC carcinogenesis and to investigate how ΔNp63 transcriptional activity as repressor or activator might be modulated in a stage‐dependent manner. These studies could unveil novel circuits linking ΔNp63 transcriptional activity and epigenetic alterations occurring in different phases of SCC development.

Another fascinating aspect of the ΔNp63‐mediated tumourigenesis is related to the functional relationship between ΔNp63 and TME. We dare to suggest that the primary oncogenic function of ΔNp63 is to activate pathways aimed to remodel ECM and TME in order to create a favourable niche for the growth and spread of malignant cells. This oncogenic function of ΔNp63 might be strictly related to the physiological function of ΔNp63 in processes such as wound healing and regeneration, in which TME modifications and ECM remodelling play a fundamental role. However, our knowledge on the functional interplay between TME and ΔNp63 in SCC as well as the role of epigenetic factors in this circuit is quite limited. Does TME modulate ΔNp63 transcriptional activity and expression? Does ΔNp63 play a role in regulating the immune landscape of SCC? Does ΔNp63 impact TME during metastatic spreading? ΔNp63/TME crosstalk could also be important in initial phases of SCC development. Genetic events altering p63 might cooperate with p53 mutations in order to trigger the initial clonal expansion of pre‐cancerous epithelial cells. These cancer‐primed cells could affect the surrounding stroma, contributing to the field cancerization, a phenomenon accounting for the frequent appearance of recurrent and multifocal tumours observed in HNSCC and lung SCC (Curtius *et al*., 2018; Dotto, 2014). How and whether ΔNp63 activity may be involved in promoting field cancerization remains an intriguing open question, which might reveal novel biomarker for cancer risk. Indeed, field cancerization can occur without any clinically detectable morphological changes, making its diagnosis difficult. In conclusion, we believe that further investigations on the oncogenic role of ΔNp63 in SCC would expand our knowledge on the pathogenesis of SCC, unveiling novel, therapeutically actionable pathways.

## Conflict of interest

The authors declare no conflict of interest.

## Author contributions

AP, GM and VG wrote the paper. VG, CF and MAP prepared the figures.
